The article "Embryonic Morphogen Nodal Is Associated with Progression and Poor Prognosis of Hepatocellular Carcinoma" was published in 2014. Journal: PLoS One.

# Embryonic Morphogen Nodal Is Associated with Progression and Poor Prognosis of Hepatocellular Carcinoma

**DOI:** 10.1371/journal.pone.0085840

**Published:** 2014-01-21

**Authors:** Jing Chen, Wen-Bin Liu, Wei-Dong Jia, Ge-Liang Xu, Jin-Liang Ma, Yun Ren, Hao Chen, Si-Nan Sun, Mei Huang, Jian-Sheng Li

**Affiliations:** 1 Department of Hepatic Surgery, Anhui Provincial Hospital Affiliated to Anhui Medical University, Hefei, China; 2 Anhui Province Key Laboratory of Hepatopancreatobiliary Surgery, Anhui Provincial Hospital Affiliated to Anhui Medical University, Hefei, China; Seoul National University, Korea, Republic of

## Abstract

**Background:**

Nodal, a TGF-β-related embryonic morphogen, is involved in multiple biologic processes. However, the expression of Nodal in hepatocellular carcinoma (HCC) and its correlation with tumor angiogenesis, epithelial-mesenchymal transition, and prognosis is unclear.

**Methods:**

We used real-time PCR and Western blotting to investigate Nodal expression in 6 HCC cell lines and 1 normal liver cell line, 16 pairs of tumor and corresponding paracarcinomatous tissues from HCC patients. Immunohistochemistry was performed to examine Nodal expression in HCC and corresponding paracarcinomatous tissues from 96 patients. CD34 and Vimentin were only examined in HCC tissues of patients mentioned above. Nodal gene was silenced by shRNA in MHCC97H and HCCLM3 cell lines, and cell migration and invasion were detected. Statistical analyses were applied to evaluate the prognostic value and associations of Nodal expression with clinical parameters.

**Results:**

Nodal expression was detected in HCC cell lines with high metastatic potential alone. Nodal expression is up-regulated in HCC tissues compared with paracarcinomatous and normal liver tissues. Nodal protein was expressed in 70 of the 96 (72.9%) HCC tumors, and was associated with vascular invasion (*P* = 0.000), status of metastasis (*P* = 0.004), AFP (*P* = 0.049), ICGR_15_ (indocyanine green retention rate at 15 min) (*P* = 0.010) and tumor size (*P* = 0.000). High Nodal expression was positively correlated with high MVD (microvessal density) (*P* = 0.006), but not with Vimentin expression (*P* = 0.053). Significantly fewer migrated and invaded cells were seen in shRNA group compared with blank group and negative control group (*P*<0.05). High Nodal expression was found to be an independent factor for predicting overall survival of HCC.

**Conclusions:**

Our study demonstrated that Nodal expression is associated with aggressive characteristics of HCC. Its aberrant expression may be a predictive factor of unfavorable prognosis for HCC after surgery.

## Introduction

Hepatocellular carcinoma (HCC) is the fifth most common malignant tumor and the second leading cause of cancer-related death in the world, with about 695,900 cancer deaths in 2008 [1]. So far, curative hepatectomy and transplantation are the most effective therapies for patients with HCC [2], but the prognosis remains poor due to high potential for metastasis and recurrence. Therefore, it is extremely needed of novel predictors to forecast prognosis and invasive phenotypes of HCC.

Embryonic morphogen Nodal, originally identified in 1994 as a member of the transforming growth factor-β (TGF-β) superfamily, was detected in the primitive ectoderm of mouse [3]. Nodal is involved in multiple biologic processes, such as induction of mesoderm and endoderm, maintenance of embryonic stem cell pluripotency, neural patterning, left-right axis specification during embryogenesis, and cancers [4], [5], [6], [7]. Nodal expression is largely restricted to embryonic tissues, and generally lost in normal adult tissues, but reemerged in human gliomas, choriocarcinoma, and cancers of breast, skin, prostate, pancreas, endometrium and ovarian [8], [9], [10], [11], [12], [13], [14], [15]. Although a recent study has reported the expression of Nodal in HCC tumor tissue [16], the function of Nodal in the progression of HCC is unclear and prognostic significance of Nodal expression is still unknown.

In the present study, we evaluated the expression of Nodal in HCC tumor tissues, paracarcinomatous tissues, normal liver tissues, 1 normal liver cell line and 6 HCC cell lines by qPCR and Western blotting to determine the relationship between Nodal expression and HCC metastatic potential. In addition, we also used immunohistochemistry to evaluate the expression of Nodal, CD34 and Vimentin in HCC tumor tissues and investigated the association of Nodal expression with angiogenesis, EMT, clinicopathological characteristics, and prognosis. Finally, we explored the role of Nodal in HCC progression, by silencing Nodal gene using small hairpin RNA (shRNA) in MHCC97H and HCCLM3 cell lines.

## Materials and Methods

### Cell culture

The normal liver cell line L02 and 6 human hepatoma-derived cell lines (Hep3B, MHCC97H, HepG2, Huh-7, MHCC97L and HCCLM3) were purchased from Liver Cancer Institute of Zhongshan Hospital, China. MHCC97L, MHCC97H and HCCLM3 were established from the same parent human HCC cell line and had a progressively increasing metastatic potential [17], [18]. Huh-7 was a non-metastatic cell line, and Hep3B and HepG2 were the cell lines with low metastatic potential. All cell lines were cultured in Dulbecco's modified Eagle's medium (DMEM) (Gibco, New York) with 10% (v/v) fetal bovine serum (FBS) (Hyclone, UT), 100 U/ml penicillin, and 100 U/ml streptomycin in a humidified 5% CO_2_ incubator at 37°C.

### Patients and tissue samples

Tumor and paracarcinomatous tissues (2 cm away from the carcinoma) for immunohistochemistry were obtained from 96 patients with HCC who had undergone curative hepatectomy between 2006.9 and 2010.6 at Department of Hepatic surgery, Anhui Provincial Hospital affiliated to Anhui Medical University. Frozen HCC tumor and corresponding paracarcinomatous tissues for Western blotting were obtained from 16 patients. Normal liver tissues were obtained from 10 patients who had received an operation due to hepatic trauma. No patient had received adjuvant therapies before surgery. The 96 patients included 78 males and 18 females with a mean age of 56.1 years (range, 25–79 years). Tumor size was measured as the largest dimension of the tumor by gross examination; Tumor differentiation was defined according to the Edmondson grading system [19]. The pathological tumor stage was defined according to the sixth edition of the tumor-node-metastasis (TNM) classification of the Inter-national Union against Cancer; All of histological diagnoses were confirmed by three experienced pathologist who were unaware of patients' clinical and laboratory data. Clinicopathologic parameters of all HCC patients were described in Table 1. Each patient had provided written informed consent prior to study participation. This study protocol was carried out with ratification by the Ethics Committee of Anhui Provincial Hospital Affiliated to Anhui Medical University and was in compliance with the ethical guidelines of the declaration of Helsinki.

**Table 1:** Clinicopathological factors and the expression of Nodal in 96 patients with HCC.

Characteristics	Number of cases	Nodal expression		?^2^	*P* value
		low	high		
*Age (years)*					
≤55	42	14	28	0.922	0.337
>55	54	12	42		
*Gender*					
Male	78	23	55	1.217	0.270
Female	18	3	15		
*Tumor size (cm)*					
≤5	60	8	52	15.318	0.000
>5	36	18	18		
*Tumor nodules*					
Single	41	9	32	0.954	0.329
Multiple	55	17	38		
*Tumor capsula*					
Complete	50	15	35	1.676	0.196
None	46	11	35		
*AFP (ng/ml)*					
≤400	47	17	30	3.850	0.049
>400	49	9	40		
*ICGR_15_ (%)*					
≤10	73	15	58	6.590	0.010
>10	23	11	12		
*HBsAg*					
Positive	78	19	59	1.563	0.211
Negative	18	7	11		
*Liver cirrhosis*					
present	81	21	60	0.352	0.553
absent	15	5	10		
*Child-Pugh grade*					
A	74	13	61	2.078	0.149
B	22	13	9		
*Edmondson grade*					
I–II	48	16	32	1.899	0.168
III–IV	48	10	38		
*TNM stage*					
I–II	43	14	29	1.182	0.277
III–IV	53	12	41		
*Vascular invasion*					
present	62	8	54	17.824	0.000
absent	34	18	16		
*Status of metastasis*					
present	26	1	25	8.203	0.004
absent	70	25	45		

The complete follow-up data were collected from all 96 patients. These patients were followed until January 6, 2013. The mean follow-up was 27.1 months (range, 2–71 months). All patients were prospectively monitored using α-fetoprotein (AFP), chest X-ray, and abdominal ultrasonography every 3–6 months after surgery. Computed tomography and/or magnetic resonance imaging were also used if necessary. The overall survival (OS) was defined as the interval between the date of surgery and the date of death or the last observation. The data were censored at the last follow-up for living patients.

### Quantitative Real-Time PCR (qPCR)

Total RNA was extracted from seven cell lines, normal liver tissues, snap-frozen HCC tumor and corresponding paracarcinomatous tissues using the TRIzol reagent (Invitrogen, USA) according to manufacturer's instruction. The quality of mRNA was evaluated by the OD260/OD280 ratio, and samples were used only when the ratio was between 1.8 and 2.0. cDNA was synthesized with oligo(dT)_18_ from 1 µg of RNA using the RevertAid First Strand cDNA Synthesis Kit (Invitrogen, USA). The sequences of Nodal-specific primers were designed as follows: forward, 5′- GGCGAGTGTCCTAATCCTGTTG -3′; reverse, 5′- CGTTTCAGCAGACTCTGGATGT-3′. For standardization of RNA quality control, expression of glyceraldehyde-3-phosphate dehydrogenase (GAPDH) in each sample was quantified by using the primer set 5′- AAGGTCATCCCTGAGCTGAAC-3′ (forward) and 5′- ACGCCTGCTTCACCACCTTCT-3′ (reverse). The PCR amplification with SYBR Premix Ex Taq (TAKARA) was performed on an ABI 7500 Real-Time instrument (Applied Biosystems) using the following conditions: 95°C for 5 sec and 60°C for 30 sec, repeated 40 cycles. A melting curve analysis was performed to monitor PCR product purity and relative gene expression data was analyzed using the 2^−ΔΔCt^ method.

### Western blotting assays

Seven cell lines in an exponentially growing phase were washed thoroughly twice with cold PBS, and then proteins from cells, normal liver tissues, snap-frozen HCC tumor and paracarcinomatous tissues were extracted using Total Protein Extraction Kit (KeyGEN, China). After centrifugation to collect lysate, protein concentration was quantified by BCA protein assay. Then, equal amounts of protein samples were concentrated and separated by running on 10% sodium dodecyl sulfate-polyacrylamide gel electrophoresis (SDS-PAGE) gel and then electrophoretically transferred onto polyvinylidene difluoride (PVDF) membranes (0.45 µm, Millipore, USA) using Trans-Blot Turbo Transfer System (Bio-Rad). Membranes were blocked with 5% non-fat milk dissolve in Tris-buffered saline containing 0.1% Tween20 (TBST) for 1 h and then incubated with primary antibody of rabbit anti-Nodal antibody (ab109317) (abcam, USA) and rabbit anti-β-actin antibody (ab133626) (abcam, USA) at 4°C overnight. After 1.5 h of incubation in horseradish peroxidase-labelled secondary antibodies (ZB-2308, ZSGB-BIO), the blots were detected using ECL western blotting kits (Pierce, USA) according to the manufacturer's instruction. The expression of β-actin was served as a loading control. The density of the bands was quantified by an Image J Software (National Institute of Heath, USA).

### Immunohistochemical staining and evaluation

Immunohistochemisty was used to detect the expression of Nodal in 10 normal liver samples, and 96 pairs of HCC tumor and corresponding paracarcinomatous tissues; CD34 and Vimentin were only examined in HCC tumor tissues. Briefly, formalin-fixed and paraffin-embedded tissues were cut into sections with a thickness of 2 µm. Sections were stained with hematoxylin and eosin (HE) for histological examination. Sections were gradually deparaffinized with xylene and alcohol. Thereafter, sections were microwave-heated for antigen retrieval in sodium citrate buffer (10 mM, pH 6.0) for 15 min, and endogenous peroxidase activity was blocked with 3% hydrogen peroxide solution for 10 min. Subsequently, mouse anti-Nodal antibody (ab55676) (abcam, USA), mouse anti-Vimentin antibody (ZM-0260, ZSGB-BIO) and mouse anti-CD34 (ZM-0046, ZSGB-BIO) antibody were respectively incubated at 4°C overnight. Following 30 min of incubation in horse-radish peroxidase-conjugated secondary antibody (PV-6000, ZSGB-BIO), sections were stained in 3, 3-diaminobenzidine tetrahydrochloride (DAB) (ZLI-9017, ZSGB-BIO) solution under microscopic observation and then counterstained lightly with hematoxylin. The positive controls were used with sections of endometrium cancer, and the negative controls were processed with PBS instead of primary antibody.

Nodal and Vimentin staining were assessed by a semi-quantitative scoring system including the intensity of staining and the proportion of stained cells [20], [21]. At low-power (40×) microscope, staining intensity of tissue sections was scored (0, no staining; 1, weak staining appearing as light yellow; 2, moderate staining appearing as yellowish-brown; 3, strong staining appearing as brown); At high-power (400×) microscope, more than five fields in one section were scrutinized, and then the percentage of positive stained cells was calculated (0, none; 1, <10%; 2, 10%–50%; 3, >50%). The final score of each section was obtained: [(score for staining intensity)×(score for percentage of positive cells)]. For category analysis, immunoreactivity of tumor cells was distinguished between high (total score≥4) and low (total score<4). CD34 antibody was used to stain vascular endothelial cells and then calculated microvessal density (MVD). The field of maximal CD34 expression was found in tumor tissues. Within this field, the area of maximal angiogenesis was selected, and microvessels were counted on a 200×magnification field [22]. The immunohistochemical results were scored by three pathologists who were blinded to clinical data.

### Plasmid extraction and RNA interference

The small hairpin RNAs (shRNA) (Shanghai Genechem, China) against Nodal were designed by inserting oligos with a hairpin loop into GV115 vector. The target sequences of Nodal shRNA (NM_018055, TAAAGACATGATCGTGGAA) were synthesized from Shanghai GeneChem Company. Bacteria containing the plasmid with Amp resistance were incubated in solid culture medium. A bacterial colony was selected and then inoculated in liquid culture medium on a vibration shaker (shaker speed 150 r/min) at 37°C overnight. Bacteria cultured overnight was harvested by centrifuging at 12000 g for 2 min. Plasmid was extracted using the QIAGEN Plasmid Mini Kit (Qiagen, Germany) according to the manufacturer's instructions, and dissolved in a suitable volume of TE buffer. We used MHCC97H and HCCLM3 cell lines in our experiments, seeding cells at 3×10^5^/ml in a 6-well plate and placed in antibiotic-free DMEM containing 10% FBS. On reaching 90% confluence, cells were transfected transiently. We then added a mixture containing 10 µl/well Lipofectamine 2000 (Invitrogen, USA), 10 µl/well plasmid, and 480 µl/well OPTI-MEM (Gibco, USA) to the plates. After 6 h at 37°C, OPTI-MEM was replaced by DMEM containing 10% FBS.

Three groups were established in this experiment: blank group (no interference), NC (negative control) group (transfected with GV115-NC shRNA, 5′-TTCTCCGAACGTGTCACGT-3′), and shRNA group (transfected with GV115-Nodal shRNA). Cells were harvested at 24, 48 and 72 h after transfection and subjected to MTT assay, flow cytometry, qPCR, Western blotting, and transwell migration and invasion assays. All experiments were performed in triplicate to confirm reproducibility. Simultaneously, a GFP (green fluorescent protein) plasmid was used to determine transfection efficiency. Cell viability was determined by MTT assay and flow cytometry.

### 3-(4, 5-dimethylthiazol-2-yl)-2, 5-diphenyltetrazolium bromide (MTT) assay

We cultured 72 h post-transfection cells (2.0×10^4^/ml, 200 µl/well) in 96-well plates with DMEM among three groups, and then added 0.5% MTT (Beyotime, China) 20 µl to each well for 4 h. The DMEM was aspirated from wells as far as possible without disturbing the cells and crystals on the plastic surface. Subsequently, 200 µl dimethyl sulfoxide (DMSO) was added to each well to dissolve crystals, and the plate agitated on a plate shaker for 10 min. Finally, optical density (OD) measurements were carried out in an enzyme-linked immunosorbent assay (ELISA) reader at a wavelength of 490 nm. The reader was calibrated to 0 absorbance using DMEM without cells.

### Flow cytometry

We collected 72 h post-transfection cells (2.0×10^5^) by centrifugation of three groups, and then suspended in 500 µl 1×Binding Buffer. Subsequently, 5 µl Annexin V-FITC and 10 µl propidium iodide (PI) (Annexin V/PI apoptosis kit, MULTISCIERNCES) were added to each sample. Samples were gently mixed and incubated at room temperature for 5 min in the dark. The cells were analyzed on a Canto-II™ reader (BD Biosciences) and data analyzed with FlowJo software (Tree Star, Ashland, OR, USA).

### Transwell migration and invasion assays

Cell migration was assayed in a transwell chamber with 24-well, 8.0-µm pore polycarbonate membrance (Corning, USA). For cell invasion assay, the same membranes were precoated with matrigel (BD Biosciences, USA). Briefly, 100 µl 1 mg/ml matrigel solution was added to the upper chamber, and then plate was immediately inverted and gelled at 37°C for 30 min in an incubator. After 72 h transfection, cells were digested and resuspended to a concentration of 1.0×10^5^/ml using serum-free DMEM with 0.1% bovine serum albumin. We seeded 200 µl cell suspensions in the upper chamber, and filled the lower chamber with 500 µl complete DMEM. The chamber was rinsed in PBS 24 h after incubation, and stained with 0.1% crystal violet for 15 min. The cells were counted using a light microscope (magnification×200). Migrated cells were averaged from 5 fields per 1 chamber and 3 chambers were used on 1 experiment.

### Statistical analysis

Statistical analyses were performed using the statistical package SPSS 13.0 (SPSS Inc., Chicago, IL). The difference in expression level of Nodal among seven cell lines and tissue samples were examined using the independent Student's *t* test. Fisher's exact tests or χ^2^ tests were performed to analyze the correlations among different protein expressions or between protein expressions and various clinicopathologic parameters. The Kaplan-Meier method was used for survival analysis, and the differences in survival were assessed by the log-rank test. The multivariate survival analysis was performed for all parameters that were significant in the univariate analysis using the Cox regression model. A *P* values less than 0.05 was considered statistically significant.

## Results

### Nodal expression in liver cell lines and snap-frozen liver tissues

To validate the up-regulation of Nodal in HCC cell lines, we used qPCR and Western blotting to detect the expression level of Nodal in 1 normal liver cell line, and 6 HCC cell lines. Western blotting analysis showed that Nodal expression was detected in MHCC97H and HCCLM3, but not in Huh-7, MHCC97L, Hep3B, HepG2 and L02 (Figure 1B). To clarify whether Nodal up-regulation was occurring at transcriptional level, qPCR analysis was performed. Results reveal that cell lines with high metastatic potential (MHCC97H and HCCLM3) showed a higher expression of Nodal in comparison with cell lines with low metastatic potential (L02, MHCC97H, Hep3B, HepG2 and Huh-7) (Figure 1A). The results demonstrate that Nodal expression was elevated at both the mRNA level and the protein level in HCC cell lines with high metastatic potential.

**Figure 1:** The expression level of Nodal mRNA and protein in liver cell lines. 1, L02; 2, MHCC97H; 3, Hep3B; 4, HepG2; 5, Huh-7; 6, MHCC97L; 7, HCCLM3. (A) Relative Nodal mRNA expression in liver cell lines measured by qPCR. (B) The expression level of Nodal protein in liver cell lines using Western blotting. Data are Mean ± SD of three replicates.

In order to determine whether the up-regulation of Nodal in HCC cell lines is clinically associated with HCC progression, 10 normal liver tissues and 16 matched pairs of tumor and paracarcinomatous tissues were analyzed by qPCR and Western blotting. As shown in Figure 2, Nodal mRNA and protein are expressed higher in HCC tumor tissues compared with paracarcinomatous and normal tissues. In addition, differences in Nodal mRNA and protein levels between paracarcinomatous tissues and normal tissues are apparent. These results also confirm the increased expression of Nodal in HCC.

**Figure 2:** The expression of Nodal protein in liver tissues. T, HCC tumor tissue; P, paracarcinomatous tissue; N, normal tissue. (A) Relative Nodal mRNA expression in liver tissues measured by qPCR. (B) The expression level of Nodal protein in liver tissues using Western blotting. Data are Mean ± SD of three replicates. * *P*<0.05.

### Immunohistochemistry of Nodal expression in HCC tumor, paracarcinomatous and normal liver tissues

To determine the role of Nodal in the clinical progression of HCC, immunohistochemical analysis was performed in 96 HCC tissue samples. Positive expression of Nodal is indicated primarily by cytoplasmic staining, with some tumor cells staining strongly, while others exhibited slight or no staining at all (Figure 3). High Nodal expression was detected in 72.9% (70/96) of HCC tumor tissues, 8.3% (8/96) in the paracarcinomatous tissues and 0 (0/10) in the normal tissues. The statistical results showed that the frequency of samples with high Nodal expression was significantly higher in HCC tissues when compared to paracarcinomatous and normal tissues, respectively (χ^2^ = 83.001, *P*<0.001; χ^2^ = 18.342, *P*<0.001, respectively). Representative immunohistochemical staining of Nodal protein in non-tumor, noninvasive and invasive tumor lesions is shown in Figure 4A. Immunohistochemical analysis suggested high Nodal expression in 0% (0/10) non-HCC patients, 47.1% (16/34) of patients with noninvasive HCC, and 79.41% (54/62) of patients with invasive HCC (*P*<0.05). The statistical results are displayed in Figure 4B. Clinicopathological analysis demonstrated that Nodal expression is significantly associated with vascular invasion (*P* = 0.000), status of metastasis (*P* = 0.004), AFP (*P* = 0.049), ICGR_15_ (*P* = 0.010) and tumor size (*P* = 0.000), but had no significant correlation with other variables (Table 1). The above results indicate that the up-regulation of Nodal may be correlated with the progression of HCC.

**Figure 3:** Immunohistochemical staining of Nodal, CD34 and Vimentin in HCC tumors. (A) HCC tumor tissue for hematoxylin-eosin staining (×400). (B) Negative Nodal expression (×400). (C) Low Nodal expression (×400). (D) High Nodal expression (×400). (E) Low Vimentin expression (×400). (F) High expression Vimentin (×400). (G) Low MVD expression (×200). (H) High MVD expression (×200).

**Figure 4:** Immunohistochemical staining of Nodal in HCC tissues and non-HCC tissues. (A) Representative images from immunohistochemistry analyses of Nodal expression in normal liver tissue (Non-HCC), HCC without invasion tissue (Non-Invasion-HCC) and HCC with invasion tissue (Invasion-HCC). (B) Percentages of high Nodal expression in Non-HCC cases, Non-Invasion-HCC cases and Invasion-HCC cases.

### Immunohistochemical expression of Nodal, CD34 and Vimentin

Angiogenesis plays an important role in the metastasis of HCC. CD34 is an antigen present in vascular endothelial cells. MVD was detected by using anti-CD34 antibody (Figure 3G and H). MVD in HCC tumors tissues ranged from 0 to 109/200×field (median, 32/200×field). Furthermore, we found that tumors with low Nodal expression show lower MVD compared with tumors showing high Nodal expression (17.6±10.7 vs. 39.5±18.4, *t* = 3.070, *P* = 0.006). Vimentin is an important characteristic of EMT, with expression observed mainly in the cytoplasm (Figure 3E and F). Among 96 patients with HCC, 58.3% of them showed high Vimentin expression. Spearman's rank correlation test was used to analyze the relationship between Nodal and Vimentin, and no relationship was found between the two indices (r = 0.198, *P* = 0.053) (Table 2).

**Table 2:** Correlation between Nodal and Vimentin expression in 96 HCC patients with HCC.

Nodal expression	Vimentin expression		*r*	*P* value
	low	high		
low	15	11	0.198	0.053
high	25	45		

### Effect of Nodal on migration and invasion in vitro

GFP fluorescence showed that plasmid Nodal shRNA was successfully transfected into MHCC97H and HCCLME3 cells. To determine the level of Nodal suppression after transfection, qPCR and Western blotting assays were performed. As shown in Figure 5, after 24, 48 and 72 h transfection, Nodal mRNA and protein expression levels significantly decreased in shRNA group, compared with blank group and NC group. In addition, no differences between blank group and NC group were apparent. These results demonstrate that Nodal shRNA effectively suppresses target gene, with the potential interference increasing gradually over 72 h after transfection.

**Figure 5:** Inhibition of Nodal by Nodal-specific shRNA in MHCC97H and HCCLM3 cells 24, 48, and 72 h after transfection, respectively. (A) Relative Nodal mRNA expression in MHCC97H cell measured by qPCR. (B) The expression level of Nodal protein in MHCC97H cell using Western blotting. (C) Relative Nodal mRNA expression in HCCLM3 cell measured by qPCR. (D) The expression level of Nodal protein in HCCLM3 cell using Western blotting. 1, control; 2, 24 h after transfection; 3, 48 h after transfection; 4, 72 h after transfection. Data are Mean ± SD of three replicates. * *P*<0.05.

To determine the role of Nodal in the progression of HCC, we performed shRNA-mediated knockdown to identify changes in high metastatic potential of HCC cells in vitro. After 72 h transfection, we performed MTT and flow cytometry assays to determine cell viability among blank group, NC group and shRNA group. OD values were not significantly different among the three groups (*P*>0.05, respectively). The results showed that the presence of only 1.4% and 2.1% cytotoxicity in MHCC97H cell compared with blank group, and 1.2% and 2.5% cytotoxicity in HCCLM3 cell. Similarly, flow cytometry results indicated that early apoptosis (Annexin V^+^ PI^−^) rates among the three groups were 0.3%, 0.7%, 2.0% in MHCC97H cell and 0.8%, 3.2%, 4.5% in HCCLM3 cell. Taken together, these results indicate that transfection does not cause severe cell damage. Next, we detected the cell migration and invasion in MHCC97H and HCCLM3 cells. The data show that the mean number of migrant and invasive cells was significantly less in shRNA group compared with blank group and NC group (*P*<0.05) (Figure 6). We have validated that Nodal expression positively correlated with cell migration and invasion in two HCC cell lines. The above results suggest that Nodal positively regulates motility and invasion of HCC cells in vitro.

**Figure 6:** Nodal suppressed migration and invasion of HCC cells in vitro. (A, B) Effect of Nodal knockdown on MHCC97H cell migration and invasion in vitro. (C, D) Effect of Nodal knockdown on HCCLM3cell migration and invasion in vitro. Data are Mean ± SD of three replicates. * *P*<0.05.

### Relationship between Nodal expression and prognosis

Kaplan-Meier survival analysis was used to assess the relationship between Nodal expression and patients' survival. The results suggested that the patients with high Nodal expression displayed a remarkably shorter OS after curative hepatectomy compared with low Nodal expression (22.0±0.3 vs. 39.9±0.7 months, respectively; *P*<0.001) (Figure 7). The 1–3-year OS rates after resection in high Nodal expression group were 83.4% and 9.7%, respectively, while in low Nodal expression group were 97.3% and 59.8%, respectively. Using the log-rank test, we found that the patients with high Nodal expression after hepatectomy have remarkably poorer OS compared with low Nodal expression (χ^2^ = 487.053, *P*<0.001).

**Figure 7:** Kaplan-Meier analysis of overall survival curves of patients with HCC according to Nodal expression. The HCC patients with high Nodal expression showed notably poorer overall survival rates than those with low Nodal expression.

Univariate analyses of prognostic factors showed that Nodal expression, gender, AFP, ICGR_15_, vascular invasion, tumor size and Edmondson grade are associated with a significant prognostic effect on OS (*P*<0.05) (Table 3). Multivariate survival analysis calculated by Cox regression using the foregoing parameters reveals that vascular invasion, tumor size and Nodal expression are independent prognostic factors for OS in patients with HCC after curative hepatectomy (*P*<0.05) (Table 4).

**Table 3:** Univariate survival analysis of OS in 96 patients with HCC.

Characteristics	OS		
	RR	95% CI	*P* value
Age (≤55 vs. >55 years)	1.498	0.943–2.378	0.087
Gender (male vs. female)	1.877	1.035–3.405	0.038
Tumor size (≤5 vs. >5 cm)	2.262	1.360–3.762	0.002
Tumor nodules (multiple vs. single)	1.110	0.701–1.757	0.657
Tumor capsula (complete vs. none)	1.526	0.961–2.421	0.073
AFP (≤400 vs. >400 ng/ml)	1.905	1.180–3.076	0.008
ICGR_15_ (≤10 vs. >10%)	1.934	1.134–3.298	0.015
HBsAg (positive vs. negative)	1.398	0.760–2.571	0.282
Liver cirrhosis(present vs. absent)	1.660	0.842–3.271	0.143
Child-Pugh grade (A vs. B)	1.456	0.777–2.730	0.241
Edmondson grade (I/II vs. III/IV)	1.700	1.056–2.736	0.029
TNM stage (I/II vs. III/IV)	1.477	0.929–2.349	0.099
Vascular invasion (present vs. absent)	2.414	1.443–4.039	0.001
Status of metastasis (present vs. absent)	1.502	0.897–2.513	0.122
Nodal (high vs. low)	3.153	1.792–5.549	0.000

**Table 4:** Multivariate survival analysis of OS in 96 patients with HCC.

Characteristics	OS		
	RR	95% CI	*P* value
Gender (male vs. female)	1.309	0.669–2.560	0.431
Tumor size (≤5 vs. >5 cm)	0.060	0.006–0.553	0.013
AFP (≤400 vs. >400 ng/ml)	1.883	0.465–7.630	0.375
ICGR_15_ (≤10 vs. >10%)	1.377	0.555–3.416	0.490
Edmondson grade (I/II vs. III/IV)	0.661	0.181–2.421	0.532
Vascular invasion (present vs. absent)	17.031	1.691–171.499	0.016
Nodal (high vs. low)	2.757	1.450–5.240	0.002

## Discussion

Previous reports suggested that Nodal was aberrantly expressed in several malignant epithelial tumors. In breast cancer progression, Nodal plays a key role in EMT, angiogenesis, invasion, migration, and apoptosis [8], [23], [24]. Furthermore, inhibition of Nodal signaling reduced tumor cell colony formation and tumorigenicity, and promoted the reversion of metastatic tumor cells toward a more differentiated, less invasive non-tumorigenic phenotype [11], [25]. The accumulated evidence suggests that high Nodal expression is common in tumor development. However, reports also suggest that Nodal plays an anti-tumorigenic role in some cancers. Zhong et al. [26]found Nodal induced apoptosis in human breast cancer cell lines. Munir and Xu [15], [27] demonstrated that Nodal inhibited proliferation and induced apoptosis in human trophoblast cells and ovarian cancer cells, respectively. These findings suggest that Nodal expression is associated with pro-tumorigenic and anti-tumorigenic effects in different pathological types of cancer. Until now, the prognostic role of Nodal in the progression of HCC has not been elucidated.

In our study, we observed that the expression of Nodal in MHCC97H and HCCLM3 metastatic cell lines was significantly higher compared with Huh-7, MHCC97L, Hep3B, HepG2 and L02 cell lines with low metastatic potential. Our findings suggest that Nodal expression is correlated with metastatic phenotype of HCC cells, and induced the metastatic phenotype of HCC in non-metastatic tumor cells. Our results are consistent with the status of Nodal expression observed in breast cancer cells [24].

Epithelial-mesenchymal transition (EMT) is a fundamental and highly conserved process underlying morphogenesis during crucial phases of embryonic development [28]. Additionally, EMT has been recognized as a potential mechanism in tumor progression, characterized by the loss or down-regulation of epithelial markers (E-cadherin) and up-regulation of mesenchymal markers (Vimentin). It is a crucial step in tumor invasion and metastasis [29]. By immunohistochemical staining, we found that Nodal expression is significantly higher in HCC tumor compared with paracarcinomatous tissues and normal liver tissues. Nodal expression is not significantly correlated with Vimentin, suggesting that Nodal has no effect on the process of EMT. However, Sun et al. [16] reported that the role of Nodal in HCC cells entailed activation of EMT through phosphorylation of Smad2/3. The discrepancy may be explained by the different origin of experimental materials, for e.g., we used anti-Nodal primary antibody from Abcam Company whereas the antibody from other company was used in other studies. Further, the small sample size in our study is limitation. The role of Nodal in EMT should be further investigated using large, randomized and multicenter studies.

In tumors, angiogenesis is considered to be one of the essential factors underlying tumor growth and metastasis [30]. Neovascularization is a common phenomenon in HCC. We evaluated the extent of angiogenesis in HCC by using CD34 antibody against vascular endothelial cell, and then quantified the MVD with a light microscope. We found that high Nodal expression is positively correlated with high MVD in HCC. The results are consistent with angiogenesis observed in breast cancer [23], showing that Nodal expression may be associated with angiogenesis.

The processes of cell migration and invasion are essential to embryonic development, and critical to immune response and tissue repair [31]. However, deregulation of these processes led to a mobile cellular phenotype, resulting in tumor metastasis. Tumor invasion is a complicated process, entailing cell-cell interactions involving extracellular matrix and accompanying biochemical processes [32]. In the present study, Nodal shRNA was successfully transfected into MHCC97H and HCCLM3 cells, and MTT and flow cytometry confirmed the transfection-associated cell damage. Subsequent, cell migration and invasion assays demonstrated that the number of migrant and invasive cells in shRNA group was significantly compared with blank group and NC group. Our results are also consistent with Nodal expression status observed in melanoma cells [11] and suggest that Nodal may promote migration and invasion of HCC cells. It is a promising molecular target for anti-Nodal therapy in HCC.

To our knowledge, our study is the first of its kind to investigate the association between Nodal expression and prognostic value in HCC. By analyzing association between Nodal expression and clinicopathological characteristics, it has been found that the vascular invasion of tumor occurs more frequently in patients with high Nodal expression compared with low Nodal expression. Results of Kaplan-Meier survival analysis suggest that patients with high Nodal expression show poor OS compared with patients showing low Nodal expression. By Cox regression analysis, high Nodal expression is an independent factor of poor prognosis of OS in patients with HCC. Therefore, the results suggest that high Nodal expression is associated with an adverse outcome in HCC, and may be used as a prognostic marker.

Nodal is a TGF-β-related embryonic morphogen, and plays an important role in normal and pathological conditions. Smad-associated Nodal signaling mediated by binding of Nodal to the Cripto-1 coreceptor and a complex of type I and type II activin receptors. The activated Smad complex induces transcription of target genes [33]. On the other hand, limited evidence involving activation of non-Smad-associated Nodal signaling is available. For example, activated p38 signaling in the anterior visceral endoderm amplified Nodal signaling during anterior-posterior axis formation [34]. Interestingly, immunohistochemical staining showed that Nodal expression was significantly increased in paracarcinomatous tissues compared with normal liver tissues, indicating that in some tumor cells Nodal expression might play a leading role in the invasion of paracarcinomatous tissues. The Nodal signaling pathway might promote the invasion and metastasis of cancer cells. Rarely, inflammation at the earliest stages of tumor progression potentially induces the transformation of incipient tumor into full-blown tumor. Tumor-associated inflammatory response had an effect on helping tumor to acquire hallmark capabilities and enhancing progression [35]. It is still unclear how the “pioneer cells” promote tumor invasion. Further experiments are therefore required to identify the precise mechanisms that regulate Nodal signaling at the cellular level in tumors.

In conclusion, our study suggests that Nodal is highly expressed in both HCC cell lines with high metastatic potential and tissues compared with their benign counterparts. Nodal does not promote EMT but induces angiogenesis. High expression of Nodal is of predictive value in HCC development and progression. We also described the inhibitory effects of Nodal shRNA transfection and show that Nodal promotes migration and invasion of HCC cells. Our findings show that Nodal acts as a novel prognostic marker and as a promising tumor-specific target in HCC progression.
